The article "Rehabilitation Training Combined with Jiaji Electroacupuncture Can Promote the Recovery of Muscle Group Function and Improve the Quality of Life in Patients with Upper Limb Peripheral Nerve Injury" was published in 2021. Journal: J Healthc Eng.

# Rehabilitation Training Combined with Jiaji Electroacupuncture Can Promote the Recovery of Muscle Group Function and Improve the Quality of Life in Patients with Upper Limb Peripheral Nerve Injury

**DOI:** 10.1155/2021/3621568

**Published:** 2021-12-20

**Authors:** Hui Li, Li Yu, Dayong Ye, Li Chang, Fengzhu Zhao, Hong Wang, Tiance Zhang

**Affiliations:** Department of Rehabilitation, The First Hospital of Qiqihar, Affiliated Qiqihar Hospital, Southern Medical University, Qiqihar 161000, Heilongjiang, China

## Abstract

This study was designed to probe into the improvement of rehabilitation training combined with Jiaji electroacupuncture intervention on patients with upper limb peripheral nerve injury. A total of 114 patients with peripheral nerve injury of upper limbs in our hospital from August 2017 to November 2019 were collected as the research participants. Among them, 59 in the control group (CG) received rehabilitation training alone, while 65 in the observation group (OG) received rehabilitation training combined with Jiaji electroacupuncture intervention. The therapeutic efficacy, Barthel index, and Fugl–Meyer assessment score, motor nerve conduction velocity, sensory nerve conduction velocity and amplitude, and quality of life (score SF-36) were compared between the two groups before and after treatment. The total effective rate of the OG was markedly higher than that of the CG. After treatment, the Barthel index, Fugl–Meyer assessment score, motor nerve conduction velocity, and sensory nerve conduction velocity and amplitude of the OG were obviously higher than those of the CG, and the SF-36 scores of the OG were higher than those of the CG in 8 dimensions. Rehabilitation training combined with Jiaji electroacupuncture intervention can dramatically promote the recovery of muscle group function and improve the quality of life of patients with upper limb peripheral nerve injury.

## 1. Introduction

Due to external trauma, upper limbs, including myelin sheath, axon, connective tissue, and peripheral nerve damage, are known as upper limb peripheral nerve injuries. Because of the compression of the upper limb nerve, ischemia, and hypoxia and the damage of other tissues around, it will affect the function of the upper limbs and lead to abnormal life and work [1–3]. However, the long-term side effects of upper limb nerve injuries and chronic neuropathic pains will influence the patients' psychological status and emotions, which greatly reduces their quality of life and treatment outcome [4, 5]. At present, there are gradually reconstructive operations clinically, but a large number of patients lose the normal function of their upper limbs after the operation. Long-term nerve injury and inability to recover will also lead to lifelong disability of patients, so further postoperative recovery is needed to cure them [6–8].

After nerve reconstruction, the regeneration of motion axis takes a long time, and the recovery and healing cycle of peripheral nerve injury of upper limbs is slow, so long-term rehabilitation training is needed to prevent muscle atrophy and degenerative diseases and gradually activate the control ability of peripheral muscles, thus accelerating the recovery of injured function of patients [9, 10]. Jiaji electroacupuncture is an important means to treat nerve injury. Electric field can promote nerve regeneration and recovery of nerve conduction function and can alleviate the degree of muscle atrophy of patients [11]. Wang et al. [12] mentioned that Jiaji electroacupuncture intervention could promote the repair process of sciatic nerve injuries in rabbits. Li et al. [13] found that the intervention might reduce the spinal cord injuries of the acute spinal cord injured rats and significantly improve motor function by reducing the spinal cord effect of nerve cell apoptosis. After peripheral nerve injuries, it will gradually lead to apoptosis of corresponding neuron cell bodies, which may be due to the fact that nutrition conduction becomes abnormal after injuries, so the bodies cannot obtain neurotrophic factors and die [14]. Therefore, in many in vitro cell and different cell injury model studies, we found that glial cell-derived neurotrophic factor and brain-derived neurotrophic factor neurons grew outward, improved the peripheral nerve injury of animal models, and reduced apoptosis and autophagy [15, 16]. Jing et al. [17] confirmed that electroacupuncture could significantly promote facial nerve regeneration by upregulating the expression of GDNF and N-cadherin in neurons, thereby inhibiting neuronal apoptosis and promoting the regeneration of peripheral facial nerve injury in rabbits. Thus, we observed the treatment plan of rehabilitation training combined with Jiaji electroacupuncture to see if it could promote treatment. The purpose of this study is to explore the effect of rehabilitation training combined with Jiaji electroacupuncture intervention on the recovery of upper limb peripheral nerve injury patients.

## 2. Data and Methods

### 2.1. Patient Data

A total of 114 patients with peripheral nerve injury of upper limbs in our hospital were collected from August 2017 to November 2019. Among them, 59 in the control group (CG) received rehabilitation training alone, including 37 males and 22 females, aged (38.2 ± 8.7), while 65 in the observation group (OG) received rehabilitation training combined with Jiaji electroacupuncture intervention, including 45 males and 20 females, aged (37.6 ± 8.3). This study was consistent with the Declaration of Helsinki and was approved by the medical ethics committee of our hospital. All patients obtained and signed an informed consent form.

### 2.2. Inclusion and Exclusion Criteria

Inclusion criteria: all patients had peripheral nerve injuries and dysfunction of upper limbs, and they had undergone surgical nerve repair operation and intended to complete treatment and follow-up investigation.

Exclusion criteria were as follows: those who were complicated with other peripheral nerve diseases; those who could not tolerate the acupuncture electromyography test; those who complicated with rheumatoid arthritis type nervous system diseases; those who complicated with other bone injury diseases; and those who had cognitive dysfunction.

### 2.3. Treatment Methods

Patients in the CG received rehabilitation training, and the medical workers should assist them with joint activity and muscle strength training. Their upper limb ability and muscle strength were improved through specific treatment tasks, and they were trained to sensation. They were trained by sensory desensitization and reeducation, and joint loosening techniques were performed regularly. Those in the OG were treated with Jiaji electroacupuncture on the basis of the CG, with C6-T1 Jiaji points, 2-inch filiform needles inclined to 1-inch bilateral points, through connected pulse electrotherapy instrument, once a day, 30 min/time, for 8 weeks.

### 2.4. Nerve Conduction Assessment

The motor nerve conduction velocity (NCV) and M wave amplitude were evaluated by stimulating the median nerve and recording the corresponding motor response of the nerve. The elbow of the subject was completely extended, the recording electrode was directly located on the motor point of the myocardium, the reference one was put on the tendon of the intercondylar joint, and the ground was located on the palm. The median nerve was stimulated on the wrist between the flexor tendon of the hand and the medial side near the chest circumference of musculus biceps. The intensity was determined by increasing the amplitude gradually until the maximum *M* wave was reached. Then, the amplitude was stimulated by 120% of this value during the test. Ten tests were carried out with a bandwidth of 10 Hz–1 kHz, and the amplitude of *M* wave was also evaluated as an indication of the motor response strength. The scanning speed was 2 s per minute, and sensitivity is 2 *μ*V per minute. The stimulation duration and rate were 0.2 s and 3 Hz, respectively.

### 2.5. Evaluation of Therapeutic Effects

Markedly effective: the pain symptoms basically disappeared, the nerve function basically returned to normal, and the nerve conduction velocity was remarkably improved; effective: the symptoms were alleviated, and the nerve function and conduction velocity were improved; ineffective: the symptoms were not alleviated, the nerve function and conduction velocity were not improved or even aggravated, and the total effective rate = (markedly effective + effective) cases/total cases × 100%.

### 2.6. Outcome Measures

The therapeutic efficacy between the two groups was counted and compared. Barthel index and Fugl–Meyer assessment score were compared before and after treatment; the former evaluated the patients' activity of daily living (ADL), 100 points in total, and the later assesses the patients' upper limb motor function, so as to evaluate the recovery of upper limb motor function, 66 points in total. Neuroelectrophysiological indexes of two groups motor nerve conduction velocity, sensory nerve conduction velocity, and amplitude were analyzed. The quality of life of patients in the two groups was observed by the SF-36 score, and the quality of life was evaluated from eight aspects: physiological function, social role, physical pain, health condition, energy, social and emotional function, and mental health, with a total score of 100 points for each item.

### 2.7. Statistical Methods

SPSS 20.0 (SPSS Co., Ltd., Chicago, the States) was used for statistical analysis. The continuous variables were expressed by the number of cases, average, and standard deviation. Both groups were compared by the independent *t*-test, the different periods between the same group were evaluated by the paired *t*-test, and the results were expressed by *t*. For classification variables, the data were expressed as the number or percentage of classification cases, detected by the chi-square test, and finally analyzed by the *X*^2^ test. *P* < 0.05 indicated that the difference was statistically marked.

## 3. Results

### 3.1. Clinical Data

By comparing the clinical data of patients in the two groups, we found that there was no remarkable difference in gender, age, time, site, and reason of injuries, nerve fracture degree, operation methods, and extent of damage between the two groups. It was comparable, as given in Table 1.

### 3.2. Therapeutic Effects

By comparing the therapeutic effects of the two groups, we found that there was no marked difference in the markedly effective and effective rates, and the total effective rate of the OG was markedly higher than that of the CG (Table 2).

### 3.3. ADL and Upper Limb Motor Function Changes

By comparing Barthel index and Fugl–Meyer assessment scores of two groups of patients, we found that two scores increased markedly, and the scores of the OG were obviously higher than those of the CG after treatment, as shown in Figure 1.

### 3.4. Neurophysiological Indicators

By comparing the neurophysiological indicators such as motor nerve conduction velocity, sensory nerve conduction velocity, and amplitude between the two groups, we found that the three after treatment were dramatically higher than those before treatment, and those of the OG were remarkably higher than those of the CG after treatment, as shown in Figure 2.

### 3.5. Quality of Life before and after Treatment

The patients' quality of life was evaluated based on the SF-36 scores of the two groups, and it was found that the scores of the OG in 8 dimensions were higher than those of the CG (*P* < 0.05), as given in Table 3.

## 4. Discussion

In this study, the therapeutic effects of the two groups were compared at first, and it was found that the total effective rate of the OG was markedly higher than that of the CG, which might indicate that the treatment scheme of rehabilitation training combined with Jiaji electroacupuncture is better than that of rehabilitation training alone. Then, we compared Barthel index and Fugl–Meyer assessment scores before and after admission. The former could better evaluate the patients' ADL, while the latter could effectively analyze upper limb disorders [18, 19]. We also discovered that the two scores of the two groups of patients increased significantly after treatment, which indicated that all of them improved their upper limb function and autonomous living function. Furthermore, we found that the scores of the OG were remarkably higher than those of the CG after treatment, which indicated that rehabilitation training combined with Jiaji acupuncture had a better recovery effect on the muscle group function of patients and could cure patients better.

Neurophysiological abnormalities can be detected by electromyography and nerve conduction research [20]. Hence, we detected electromyography indexes including motor nerve conduction velocity, sensory nerve conduction velocity, and amplitude before and after treatment in both groups. All the three in the OG were markedly higher than those in the CG after treatment, which also verified that rehabilitation training combined with Jiaji acupuncture therapy had better therapeutic advantages. He et al. [21] reported that electroacupuncture could ensure and improve the continuity between peripheral and central nerve, thus shortening the repair process of the damaged nerve, providing the basis for regeneration, and recovering motor conduction well. Many studies have mentioned that the treatment of peripheral nerve injury by electrical stimulation has a good therapeutic effect. For example, Yu et al. [22] found that electrical stimulation could enhance nerve regeneration and functional recovery, and the implementation of electrode point and 1/4 circle contact on the sciatic nerve resection model could significantly improve sciatic nerve function index, compound muscle action potential, and motor nerve conduction velocity scores and could better promote sciatic nerve regeneration and reduce muscle atrophy, with less mechanical damage to nerve trunk. Pan et al. [23] studied that electrical stimulation could remarkably treat peripheral neuropathy caused by diabetes, reduce the apoptosis of sciatic nerve cells in diabetic rats, and prevent sciatic nerve injury by inhibiting the occurrence of endoplasmic reticulum stress. At the end of the study, we counted and compared the quality of life of the two groups of patients. Because of severe neuropathic pain and the possibility of disability, the quality of life of those with peripheral nerve injury of upper limbs was not high [23]. Our research shows that the quality of life of patients with combined treatment was remarkably higher than that of those with rehabilitation training alone.

## 5. Conclusion

To sum up, rehabilitation training combined with Jiaji electroacupuncture can significantly promote the recovery of muscle group function and improve the quality of life of patients with upper limb peripheral nerve injury.

However, there are some shortcomings in our research. First of all, there are some differences in the surgical methods for patients, but the research on porcelain fracture has not explored this. Second, we have not further explored the specific mechanism of improvement, so we hope to carry out corresponding animal experiments to support our conclusions. At the moment, there are some new therapies for peripheral nerve reconstruction and recipient nerve regeneration, such as using allogeneic transplantation or other transplantation materials. It is also found that patients have better nerve regeneration after operation, the biological activity of cells has been improved, the inhibition of apoptosis has been suppressed, and the immune rejection is less [24], which may also become the focus of our future research.

## Figures and Tables

**Figure 1:** Changes of ADL and upper limb motor function. (a) The Barthel index of both groups after treatment is significantly higher than that before treatment and that of the observation group is significantly higher than that of the control group after treatment. (b) After treatment, the scores of Fugl–Meyer assessment scale in the two groups are significantly higher than those before treatment, and the observation group is significantly higher than that in the control group.

**Figure 2:** Changes of neurophysiological indicators before and after treatment. (a) Motor nerve conduction velocity of two groups of patients after treatment is significantly higher than that before treatment and that of the observation group is significantly higher than that of the control group after treatment. (b) Sensory nerve conduction velocity of the two groups after treatment is significantly higher than that before treatment, and the observation group is significantly higher than that of the control group after treatment. (c) After treatment, the amplitude of patients in the two groups is significantly higher than that before treatment and that in the observation group is significantly higher than that in the control group after treatment.

**Table 1:** Clinical data sheet.

	Control group (*n* = 59)	Observation group (*n* = 65)	*X* ^2^/*t*	*P*
Gender				
Male	37 (62.71)	45 (69.23)	0.587	0.444
Female	22 (37.29)	20 (30.77)	0.695	0.393
Age (years)	38.2 ± 8.7	37.6 ± 8.3		
Injury time (h)	5.09 ± 1.17	5.04 ± 1.19	0.236	0.814
Injury site			0.874	0.646
Radial nerve	24 (40.68)	29 (44.62)		
Ulnar nerve	17 (28.81)	27 (41.54)		
Median nerve	18 (30.51)	19 (29.23)		
Cause of injuries			3.917	0.271
Traffic accidents	16 (27.12)	13 (20.00)		
Incised wound	9 (15.25)	12 (18.46)		
Hinge rolling injury	20 (33.90)	31 (47.69)		
Puncture wound	14 (23.73)	9 (13.85)		
Degree of nerve rupture			0.700	0.403
Incomplete fracture	31 (52.54)	39 (60.00)		
Complete fracture	28 (47.46)	26 (40.00)		
Operation modes				
Repair of neurological defect	34 (57.63)	40 (61.54)	0.282	0.869
Neuroanastomosis	10 (16.95)	9 (13.85)		
Neurolysis	15 (25.42)	16 (24.61)		
Extent of damage			0.955	0.328
Moderate injury	25 (42.37)	22 (33.85)		
Severe injury	34 (57.63)	43 (66.15)		

**Table 2:** Therapeutic effect table.

	Control group (*n* = 59)	Observation group (*n* = 65)	*X* ^2^	*P*
Markedly effective	18 (30.51)	27 (41.54)	1.627	0.202
Effective	29 (49.15)	33 (50.77)	0.032	0.857
Ineffective	12 (20.34)	5 (7.69)	4.181	0.041
Total effective rate	47 (79.66)	60 (92.31)		

**Table 3:** SF-36 scoring results table.

	Control group (*n* = 59)	Observation group (*n* = 65)	*X* ^2^	*t*
Physiological function	63.56 ± 17.25	70.26 ± 16.93	2.181	0.031
Mental health	54.26 ± 14.33	66.52 ± 16.23	4.440	<0.001
Somatic pain	64.64 ± 15.36	74.84 ± 12.75	4.037	<0.001
Emotional function	60.62 ± 15.38	68.20 ± 17.52	2.549	0.012
Energy	51.53 ± 13.92	57.42 ± 13.55	2.386	0.019
Social role	51.37 ± 22.15	61.76 ± 16.64	2.970	0.004
Health status	54.33 ± 12.85	62.39 ± 11.24	3.725	<0.001
Social function	52.46 ± 13.65	58.77 ± 12.94	2.642	0.009

## Data Availability

The datasets used and/or analyzed during the current study are available from the corresponding author upon request.
